The article "Decrease expression and clinicopathological significance of miR-148a with poor survival in hepatocellular carcinoma tissues" was retracted in 2016. Reasons: misconduct by an author; plagiarized text; plagiarized images; compromised peer review.

# Decrease expression and clinicopathological significance of miR-148a with poor survival in hepatocellular carcinoma tissues

**DOI:** 10.1186/s13000-015-0371-4

**Published:** 2015-08-07

**Authors:** Hossein Ajdarkosh, Masoomeh Dadpay, Emad Yahaghi, Elham Rostami Pirzaman, Amir Farshid Fayyaz, Ebrahim Khodaverdi Darian, Aram Mokarizadeh

**Affiliations:** Gastrointestinal and Liver Disease Research Center (GILDRC), Firoozgar Hospital, Iran University of Medical Sciences, Tehran, Iran; Department of Pathology, Imam Reza Hospital, AJA University of Medical Sciences, Tehran, Iran; Baqiyatallah University of Medical Sciences, Tehran, Iran; Department of Biotechnology and Nanotechnology, Zanjan University of Medical Sciences, Zanjan, Iran; Department of Legal Medicine, AJA University of Medical Sciences, Tehran, Iran; Young Researchers and Elite Club, Karaj Branch, Islamic Azad University, Karaj, Iran; Cellular & Molecular Research Center, Kurdistan University of Medical Sciences, Sanandaj, Iran

## Abstract

**Background:**

Hepatocellular carcinoma (HCC) is a leading cause of cancer-related death worldwide, mainly due to its high rates of postoperative recurrence and metastasis. Please remove, it currently ranks as the third most common cause of cancer-related deaths. MiRNAs are a set of small, single-stranded, non-coding RNA molecules that negatively regulate gene expression at the post-transcriptional level. In this study, we demonstrated the down-regulation of miR-148a in HCC and non-cancerous tissues using qRT-PCR.

**Methods:**

Ninety six HCC samples and their noncancerous normal liver tissues were collected. Total mRNA including miRNA was extracted, and miR-148a expression was determined using qRT-PCR. Furthermore, the correlation between the miR-148a expression and clinicopathological parameters was investigated.

**Results:**

The result showed that reduction of miR-148a expression was associated with TNM stage, metastasis, and number of tumor nodes. Multivariate Cox proportional hazards model analysis showed that low expression of miR-148a was independently associated with recurrence of HCC in the current study. Moreover, our result showed that lower expression in tumor tissues in comparison with corresponding normal control tissues.

**Conclusion:**

Down-regulation of miR-148a is related to HCC carcinogenesis and deterioration of HCC. MicroRNA-148a may act as a suppressor miRNA of HCC, and it is therefore a potential prognostic biomarker for HCC patients.

## Background

Hepatocellular carcinoma (HCC) is known as the sixth common malignancies all over the world, and is the second cause of cancer-related mortality [1, 2]. In 2012, 782,000 new cases and 746,000 deaths from HCC have been reported. Although the clinical staging have used in clinical decision, but improvement of molecular mechanism can be useful to clarify the role of new markers in the treatment and prognosis of HCC [3].

MicroRNAs (miRNAs) are a class of small non-coding RNAs [4]. It has been reported that dysregulation of miRNA expression profiles presented in HCC cancer and indicated that miRNAs can be beneficial markers for HCC progression and clinical course [5–9]. MiRNAs are as either oncogenes or tumor suppressors in human carcinogenesis [10]. The mature members of miR-148/152 family have been proved to be expressed in different tumors that paly significant role in development and tumorigenesis.

In addition, down-regulation of MiRNA-148a, was previously shown in many types of cancers [11, 12]. These studies suggested that MiRNA-148a has prognostic value in clinical evaluations and can act as tumor-suppressor miRNAs. In current study, we evaluated the clinical significance of miR-148a in HCC patient and its association with clinicopathological features.

## Methods

### Patients

This retrospective study, we investigated 96 patients diagnosed with HCC who had undergone surgery at Tehran hospitals between May 2008 to September 2013. Moreover, adjacent noncancerous liver tissues were at least 2 cm away from the tumor node, were obtained from 30 patients who underwent surgery for reasons other than malignancy. Tissues were snap frozen in liquid nitrogen after surgical resection until use. The clinicopathological features of the patients are summarized in Table 1. This study was approved by the Research Ethics Committee. In addition, the diagnosis and the histologic grade were confirmed by two pathologists.

**Table 1:** Relationship between the miR-148a expression and clinicopathological features of patients with HCC (X^−^ ± S)

Characteristic	Number	miR-148a expression		
		2-Δcq	T	*P* value
Gender				
Male	55	0.71 ± 0.40	0.561	0.712
Female	41	0.85 ± 0.58		
Age				
≤60	42	0.74 ± 0.71	−0.579	0.462
>60	54	0.95 ± 0.47		
Tumor diameter (cm)				
≤5	55	0.84 ± 0.43	3.734	0.316
>5	47	0.80 ± 0.58		
Vein invasion				
Negative	81	0.77 ± 0.43	−0.273	0.131
Positive	20	0.80 ± 0.55		
With cirrhosis				
Negative	18	0.71 ± 0.45	−0.236	0.621
Positive	78	0.80 ± 0.52		
Metastasis				
Yes	46	0.82 ± 0.46	−1.767	0.021
No	50	1.32 ± 0.63		
TNM stage				
I + II	41	1.53 ± 0.41	4.126	0.042
III + IV	55	0.86 ± 0.34		
Differentiation				
Well	4	0.71 ± 0.32	−0.842	0.412
Moderate	77	0.85 ± 0.47		
Poor	15	0.62 ± 0.34		

### RT-qPCR assay

Total RNA was purified using TRIzol® reagent (Invitrogen Life Technologies, Carlsbad, CA, USA). Moreover, we applied a miRNA Reverse Transcription kit (Invitrogen Life Technologies) to convert RNA into cDNA.

RT-qPCR was carried out using a miRNA qPCR Detection kit (GeneCopoeia, Rockville, USA) by system of thermocycler. We used the comparative cycle threshold (CT) method to calculate changes in expression. The relative amount of miR-148a was normalized with U6 gene as internal reference. In addition, the 2^−ΔΔCt^ method was used to evaluate the expression level of miR-148a in cancer and normal samples were evaluated.

### Statistical analysis

SPSS software 20.0 (Chicago, IL, USA) was used for statistical analysis. The chi-square test was used to assess miR-148a expression with respect to clinicopathological factors. Kaplan-Meier Survival method was used to evaluate the association between miR-148a and recurrence *P* < 0.05 was considered to indicate a statistically significant difference.

## Results

Significantly decreased expression of miR-148a was observed in the HCC tissues than in the adjacent normal hepatic tissues. ROC analysis was used to evaluate the diagnostic value of miR-148a. The area under the curve (AUC) of miR-148a was 0.837 (95 % CI 0.782 - 0.954, *P* < 0.035). In addition, the median 2-Δcq 0.93 was calculated as the cut-off value of miR-148a. As shown in Fig. 1, the sensitivity and specificity were calculated to be 80 % and 62.2 %, respectively. Furthermore, results suggested that expression of miR-148a in advanced stages (III and IV) was remarkably low than that in early stages (I and II), (*P* = 0.042). Low expression was also associated with metastasis (*P* = 0.021). However, miR-148a expression was not associated with sex (*P* = 0.712), age (*P* = 0.462), Tumor diameter (P = 0.316), liver cirrhosis (0.621), and differentiation (*P* = 0.412), (Table 1). The result indicated that the patients with low expression of miR-148a had a longer time-to-recurrence when compared with low expression patients (1.47 ± 0.42; 2.87 ± 0.64 mean ± SD), Nevertheless, there was no significant difference between two groups (*P* = 0.417). Multivariate Cox proportional hazards model analysis showed that low expression of miR-148a was independently associated with recurrence of HCC (HR = 2.68; 95 % CI: 1.416-8.367, *P* = 0.026).

**Fig. 1:** The area under the curve (AUC) of miR-148a with the sensitivity and specificity were calculated to be 80 % and 62.2 %, respectively

## Discussion

This study aimed to evaluate the clinical significance of miR-148a in HCC patient and its association with clinicopathological features. Significantly decreased expression of miR-148a was observed in the HCC tissues than in the adjacent normal hepatic tissues. This finding suggested that miR-148a could play a key role in suppression and progression of tumor. The ROC curve suggested a moderate diagnostic value of miR-148a in HCC with the AUC as 0.837. The results of our study, together with those reported previously, suggested that miR-148a plays a critical role as oncogene or tumor suppressor in many tumors [11–14]. On the other hand, Zhao et al. reported that up-regulation of miR-148b induced the apoptosis and cell-cycle arrest of pancreatic cancer cells by targeting AMPKa1 [13]. In addition, miR-148b was reported to regulate the metastasis of hepatocellular carcinoma cells through targeting CCK2R [13].

Concerning the relationship between expression of miR-148a and clinicopathological features, the expression level of miR-148a in advanced stages (III and IV) was remarkably low than that in early stages (I and II), (*P* = 0.042). In addition, low expression was also associated with metastasis (*P* = 0.021). It has been previously reported that miR-148b might be linked to tumor invasion and progression in many kind of tumors, in the present study, similar trend was observed [12, 15–20]. However, Cuk K et al. found that miR-148b is significantly upregulated in the plasma of breast cancer patients and may be used for the efficient diagnosis [21]. Previously, miR-148b was suggested to be upregulated in ovarian cancer, and its upregulation may be involved in the early stage of ovarian carcinogenesis [22]. Recently, Gailhouste et al. [23] showed that miR-148a could promote the hepatospecific phenotype, and acted as a tumor suppressor by targeting the c-Met oncogene. It was found that overexpression of miR-148a led to a notable inhibition of the invasive properties of hepatocellular carcinoma cells, whereas silencing of miR-148a promoted hepatocellular carcinoma cell invasion [23]. These controversial results of miR-148a in cancer development may reflect the diverse roles of miR-148a in different types of cancer. In the present study, we identified that miR-148a is a predominantly downregulated miRNA in HCC tissues compared with normal liver tissues by using qRT-PCR assay, suggesting that miR-148a might be implicated in tumorigenesis. Mentioned studies and this current study, point in the same direction, that there is a remarkable association between miR-148a and the infiltration of tumor cells, migration, invasion and metastasis of tumors. Hence, it may be useful to clinically evaluate miR-148a expression for the prediction of metastasis and deterioration in HCC patients.

In the next step, we evaluate the association between miR-148a and recurrence. The result suggested that the patients with low expression of miR-148a had a longer time-to-recurrence when compared with low expression patients (1.47 ± 0.42; 2.87 ± 0.64 mean ± SD), Nevertheless, there was no significant difference between two groups (*P* = 0.417). A larger cohort is required to evaluate the relationship between miR-148a and tumor recurrence in future studies. The mechanisms whereby miR-148a was down-regulated in the advanced stages of HCC could be associated with diverse target genes and pathways involved. Therefore further investigation is needed to clarify such mechanisms.

Multivariate Cox proportional hazards applied in the present study which suggested that low expression of miR-148a was independently associated with recurrence of HCC (HR = 2.68; 95 % CI: 1.416-8.367, *P* = 0.026).

## Conclusions

In conclusion, the findings indicated that down-regulation of miR-148a is related to HCC carcinogenesis and deterioration of HCC. MicroRNA-148a may act as a suppressor miRNA of HCC, and it is therefore a potential prognostic biomarker for HCC patients.
